The article "Ferroptosis: A Novel Therapeutic Direction of Spinal Cord Injury" was retracted in 2023. Reasons: signs of a paper mill; suspected computer-generated content; unreliable results or conclusions; concerns about the data.

# Ferroptosis: A Novel Therapeutic Direction of Spinal Cord Injury

**DOI:** 10.1155/2022/7906218

**Published:** 2022-07-12

**Authors:** Qianlong Zhao, Feifei Liu, Bangyu Zhou, Hongzhi Liu, Xiaowei Wang, Shaobo Li

**Affiliations:** ^1^School of Clinical Medicine, Dali University, China; ^2^Department of Spine Surgery, The First Affiliated Hospital of Dali University, China; ^3^Teaching and Research Department of Surgery, School of Clinical Medicine, Dali University, China

## Abstract

An injury to the spinal cord results in a crucial central nervous system event that further causes irreversible impairment or loss of motor, autonomic, and sensory functions. A progressive pathophysiological cascade following spinal cord injury (SCI) includes ischemia/reperfusion injury, oxidative stress, proapoptotic signaling, peripheral inflammatory cell infiltration, and glutamate-mediated excitotoxicity, and regulated cell death. These complex pathological and physiological changes continue to cause cell injury over the long-term and severely limit the efficacy of clinical treatment strategies in restoring the injured nervous system. Ferroptosis is a nonapoptotic, iron-regulated kind of cell death that has recently been discovered. It is distinguished by iron overload-induced toxic lipid peroxidation associated with mitochondrial morphological changes during the cell death process. For example, after SCI, iron overload activates the reactive oxygen species generation, dysregulation of glutathione/glutathione peroxidase 4 (GSH/GPX4) metabolism, and accumulation of lipid peroxides, which cause lipid membrane deterioration and ferroptosis. Conversely, knockout or differential expression of key genes and application of lipid peroxidation inhibitors and iron chelators (e.g., deferoxamine) (e.g., SRS-16-86) can block ferroptosis and promote neuronal repair for functional recovery after SCI. Although the findings of numerous investigations have been confirmed the importance of ferroptosis in several human neurologic sicknesses and its potential in SCI, the mechanism of ferroptosis and its application in SCI has not been elucidated. This review highlights current ferroptosis research and its impact on SCI, as well as the key molecular mechanism of ferroptosis in promoting the recovery from SCI. Understanding ferroptosis' process and function in SCI could provide useful insight into the treatment and avoidance of such a destructive injury.

## 1. Introduction

An injury to the spinal cord is a severely disabling and fatal clinical disease and is associated with a high economic burden. The global incidence of SCI has continuously grown over the past 30 years. The prevalence of SCI varies from 236 to 1,298 people per million in different countries. Every year, 250000–500000 individuals have diagnosed with SCI globally [1]. In clinical practice, the treatment of SCI mainly includes methylprednisolone administration, surgical decompression, supportive care, and physical rehabilitation. However, these treatments have a suboptimal effect [2], and despite a lot of research on restoring the spinal cord defect and nerve function after SCI, there are no effective measures to cure SCI. It has been suggested that the regulation of the execution of cell lethal procedures after SCI at cellular and molecular levels may create avenues for a better therapeutic effect [3]. In the process of regulated cell death (RCD) [4], various types of lethal sequences have a varying extent of the effect on the progress and therapeutic effect of SCI. Recently, the most extensively researched apoptosis, pyroptosis, necroptosis, autophagy, and ferroptosis are the five types. Every type has its molecular uniqueness mechanism [5].

The article "Ferroptosis: A Novel Therapeutic Direction of Spinal Cord Injury" was retracted in 2023. Reasons: signs of a paper mill; suspected computer-generated content; unreliable results or conclusions; concerns about the data.

Ferroptosis is a new type of RCD, which involves the activation, expression, and regulation of a series of genes [6]. Early studies on ferroptosis mainly focus on the field of the tumor, and the function of ferroptosis in tumors is related to their malignant transformation, evolution, and drug resistance development [7]. The results of accumulating research on ferroptosis have suggested that ferroptosis may be generated in a variety of ways by tumor cells and is associated with ischemia/reperfusion-induced heart and liver damage, acute kidney failure, and central nervous system diseases [8, 9].

In recent years, the role of ferroptosis in spinal cord injury has attracted wide attention, and the use of small molecular compounds has been shown to inhibit this process and encourage the reestablishment of neuronal function [10]. This opens new avenues to explore a cure for SCI. This article reviews recent studies on ferroptosis and SCI to provide new opportunities and potential for further research.

## 2. The Basic Mechanism of Ferroptosis

The word “ferroptosis” was coined by American researchers Stockwell and Dixon in 2012 who found that after-care for human NRAS mutant HT-1080 fibrosarcoma cells with the small molecular probes Erastin and RSL3 caused iron-dependent lipid peroxidation accumulation and eventually led to new regulatory cell death [6].

The ferroptosis is caused by iron overload, lipid peroxidation, and the accomplishment of downstream cascade procedures [6], whereas the regulatory mechanism involves the SCT/GSH/GPX4 pathway [11] in addition to the transsulfuration and mevalonate pathways [9]. Ferroptosis triggers could be from extrinsic or intrinsic pathways [12]. Ferroptosis activation by the external route is through interfering with membrane transporters, as an example glutamate/cystine transporters. Alternatively, the iron transporters serotransferrin and lactotransferrin can be activated. Ferroptosis activation by the natural route is through the intracellular antioxidant enzymes are blocked (such as glutathione peroxidase GPX4) [5].

The article "Ferroptosis: A Novel Therapeutic Direction of Spinal Cord Injury" was retracted in 2023. Reasons: signs of a paper mill; suspected computer-generated content; unreliable results or conclusions; concerns about the data.

Unlike other types of RCD, for example, apoptosis, necrosis, the morphology, molecular biological, and genetic characteristics of ferroptosis are distinct. One of the features of ferroptosis is the decrease or the obliteration of mitochondrial cristae along with the transport or shrinkage of the outer mitochondrial membrane [6, 13]. Phospholipid peroxidation causes cell death via ferroptosis, iron loading, increased reactive oxygen species (ROS) levels, and phospholipids containing polyunsaturated fatty acid chains (PUFA-PLs). Excess lipid peroxidation destroys the lipid membranes and ultimately induces ferroptosis via a cascade wherein cellular antioxidant systems, such as cystine uptake, glutathione synthesis, GPX4 functioning, and lipid peroxidation, break down [6, 11]. This pattern of cell death is not affected by the inhibitors of apoptosis, necrosis, or autophagy [6] and is rather affected by inhibiting or knocking out key genes to change the genetic phenotype. Application of lipid antioxidants, such as SRS16-86, Lip-1, or vitamin E, as well as an iron chelator in SCI, can inhibit ferroptosis through different pathways, as displayed in Figure 1.

After spinal cord injury, the ion disorder leads to an abnormal increase in the level of Fe^3+^, which binds to the ferritin receptor, enters the cell, and then, enters the endosome. STEAP3 reduces Fe^3+^ to Fe^2+^ within the endosome. Free iron (Fe^2+^) is transported from the endosome to the cytoplasm through DMT1, thus forming a “labile iron pool.” Some Fe^2+^is oxidized to Fe^3+^by CP or HEPH and carried out of the cell by SLC40A1, and some are stored in ferritin by PCBP1. Under the influence of some factors, NCOA4 mediates ferritinophagy and releases free iron in ferritin, and the abnormal iron homeostasis finally induces the production of ROS. Cystine and glutamate were reverse-transported through the x_c_^−^ system on the cell membrane at 1 : 1. Cystine entering the cell is shrunk down to the cysteine for the synthesis of GSH. The transsulfuration process can augment cysteine levels. With the assistance of GSH, GPX4 reduced PL-OOH to the corresponding alcohol or free lipid hydrogen peroxide. PUFAs rich in AA and ADA are regulated by ACSL4 and LPCAT3 to form AA-PE and ADA-PE, respectively. Then, PL-OOH is formed under the catalysis of iron-containing enzymes (particularly lipoxygenase LOX-15), which causes lipid peroxidation and induces ferroptosis.

The article "Ferroptosis: A Novel Therapeutic Direction of Spinal Cord Injury" was retracted in 2023. Reasons: signs of a paper mill; suspected computer-generated content; unreliable results or conclusions; concerns about the data.

## 3. The Essential Processes of Ferroptosis

### 3.1. Iron Metabolism Pathway and Ferroptosis

Iron is an important micronutrient in the body and participates in many complex biochemical reactions. In the central nervous system, cells contain a certain level of iron to be involved in oxygen transport, oxidative phosphorylation, myelination, and the synthesis and metabolism of neurotransmitters. Oxidation and alteration of lipids, proteins, carbohydrates, and DNA can occur when iron homeostasis is disrupted through the production of hydroxyl radicals, which can lead to cellular damage [14].

The iron present in the human body can be classified into free iron (Fe^2+^ and Fe^3+^) and bound iron; bound iron exists mainly in the kind of ferritin [contains ferritin light chain (FTL) and ferritin heavy chain 1 (FTH1)], for example, hemoglobin and iron-sulfur nanocluster, and free iron is also called unbound iron, which is mostly present in heme or noniron–sulfur nanoclusters [8, 9].

The accumulation of iron is an essential part of ferroptosis [15]. The free Fe^3+^ in circulation usually binds to transferrin and locates in endosomes after entering the cell through transferrin receptor 1 (TFR1); in endosomes, the ferrireductase six-transmembrane protein of prostate 3 (STEAP3) also facilitates this process by reducing Fe^3+^to Fe^2+^ before transport through DMT1. Fe^2+^ is either released from endosomes into the cytoplasmic “labile iron pool (LIP)” under the auspices of divalent metal transporter 1 (DMT1, also known as SLC11A2) or transferred through poly (RC)-binding protein1 (PCBP1) and stored in ferritin [16]. Ferritin may be broken down by lysosomes to liberate unbound iron and the inhibition of nuclear receptor coactivator 4- (NCOA4-) mediated ferritinophagy, which is a selective autophagy in lysosomal degradation of intracellular ferritin, can reduce free Fe^2+^, and ultimately limit ferroptosis [17, 18]. Fe^2+^with redox activity in the LIP catalyzes the production of ROS, including superoxide radicals (•O ^−^) and hydroxyl radicals (•OH) by Fenton reaction, which provides highly reactive free radicals for lipid peroxidation to promote ferroptosis [19].

However, loosely connected iron or iron complexes (heme or [Fe-S] cluster) are the basic reaction of numerous enzymes' components; these enzymes participate in the formation of LOX, cytochrome P450, xanthine oxidase, NADPH oxidases, and mitochondrial complex I and III, among others; some of these enzymes (e.g., catalase and peroxidase) are also involved in the decomposition of ROS [20]. Finally, ferrous oxidases, such as ceruloplasmin (CP) or hephaestin (HEPH), reoxidize excess Fe^2+^to Fe^3+^, and iron, are excreted from the cell by the iron-efflux protein solute carrier family 40 member 1 (SLC40A1/ferroportin1/FPN) [16].

The article "Ferroptosis: A Novel Therapeutic Direction of Spinal Cord Injury" was retracted in 2023. Reasons: signs of a paper mill; suspected computer-generated content; unreliable results or conclusions; concerns about the data.

Therefore, it can be seen that reducing iron storage by increasing iron intake or reducing iron output and promoting ferritin self-degradation can lead to intracellular iron overload, thus resulting in oxidative stress and ferroptosis. Furthermore, new research has discovered that iron overload is caused by several different types of iron complexes (e.g., ferric chloride, heme, hemin, or ammonium ferrous sulfate), which induces atypical pathways of ferroptosis [9].

The significance of iron in ferroptosis has been proposed and widely discussed since the first report on ferroptosis, and notably, if ferroptosis is indeed a controlled procedure, then the gene products related to iron uptake and/or release may also be important participants in the process, such as iron-responsive element-binding protein 2 (IREB2), which is the most important factor in iron metabolism and affects the uttering of TFRC, ISCU, FTH1, and FTL during ferroptosis [16, 21]. Heme oxygenase 1 (HMOX1) with its antioxidant activity moderately activates protection against ferroptosis, whereas overactivation of HMOX1 can catalyze the degradation of heme to ferrous iron, biliverdin, and carbon monoxide, which would, in turn, promote ferroptosis by increasing the LIP [11]. In related studies, ferroptosis can be suppressed using an iron chelator, such as deferoxamine (DFO) [22], DFP [23], and BPS [24], thus providing a potential therapeutic strategy for SCI.

### 3.2. Lipid Metabolism and Peroxide Accumulation

Lipid peroxidation is closely associated with ferroptosis occurrence. Long-chain PUFAs rich in arachidonic acid (AA) and adrenoyl (ADA) are the primary substrates for lipid peroxidation, which cause serious damage to the plasma membrane and affect the integrity of cells and their function. In this process, lipid peroxidation products can be formed by autooxidation, free radical chain reactions, and enzyme catalysis [25].

Hydroxyl radical is the most chemically active ROS, and the Fenton and Fenton-like reactions (which are both central to advanced oxidation technologies to remediate organic pollutants) are its main source. Hydroxyl radicals (OH^•^) can extract hydrogen from the polyunsaturated fatty acids and form carbon-centred lipid-free radicals, which can readily and rapidly react with oxygen to form PL peroxide radicals (PL-OO•). PL-OO•, in turn, absorbs the hydrogen of the adjacent polyunsaturated fatty acids to form PL-OOH and a new PL radical, thus spreading the chain reaction [11]. The autooxidation of lipids can be automatically catalyzed because the O-O bond of PL-OOH can be broken in the presence of Fe^2+^, thus converting it to PL alkoxy (PL-OO•), which also contributes to the spread of free radical chain reaction [26]. However, the reaction can terminate if a chain-breaking antioxidant, such as vitamin E, is present. Enzymatic lipid peroxidation can be carried out through cyclooxygenase (COX), cytochrome P450 oxidoreductase (POR), NAPDH oxidase (NOX), and lipoxygenase (LOX).

The article "Ferroptosis: A Novel Therapeutic Direction of Spinal Cord Injury" was retracted in 2023. Reasons: signs of a paper mill; suspected computer-generated content; unreliable results or conclusions; concerns about the data.

There are mainly two kinds of cyclooxygenases in the human body, COX-1 and COX-2 [27], and their active products are mainly aliphatic alcohols and not lipid hydroperoxides. By providing electrons to the downstream effectors, such as CYPs, POR can directly participate in lipid peroxidation [28]. NOX-specific inhibitors (e.g., DPI and GKT137831) can significantly inhibit elastin-induced ROS production and ferroptosis in some cells, suggesting the involvement of NAPDH oxidase in ROS production during lipid peroxidation [6]. Lipoxygenases are nonheme iron-containing dioxygenases that catalyze the insertion of oxygen into PUFAs at the bis-allylic position in the nonbilayer phospholipid arrangement to produce various lipids and hydrogen peroxides [29]. There are six human isomers in the lipoxygenase family, namely, ALOXE3, ALOX5, ALOX12, ALOX12B, ALOX15, and ALOX15B [29]. The polyunsaturated fatty acids AA and AdA are esterified into membrane phospholipids to produce phosphatidylethanolamine-linked AA (PE-AA) and PE-AdA, respectively, under the control of two lipid metabolic enzymes, namely, Acyl-CoA synthetase long-chain family member 4 (ACSL4) and lysophosphatidylcholine acyl-transferase 3 (LPCAT3) [30, 31]. ACSL4 and LPCTA3 can induce cell membrane to be empathetic to PUFAs (such as AA and AdA) and lipoxygenase (LOX), particularly 15-lipoxygenase (15- LOX) [32]. In the presence of LOX, PE-AAs and PE-AdAs, which are rich in PUFAs, are oxidized into their respective lipid peroxidation products PE-AA-O-OH or PE-AdA-O-OH, thus resulting in ferroptosis [25, 33]. If the ACSL4 gene is knocked out or LPCAT3 is absent, some nonneuronal cells will develop significant resistance to ferroptosis [30, 31]. In addition, lipid peroxidation reportedly plays an important last stage of the process of ferroptosis [34]. Even so, the descending enforcement mechanism is ambiguous, and lipid hydrogen peroxide can be broken down into reactive toxic aldehydes (e.g., 4-HNEs or MDAs). These catabolic substances promote ferroptosis by covalently modifying proteins and nucleic acids that are involved in basic cellular processes and by forming covalent adducts in reaction with lipid membranes to regulate many signaling processes [35]. Furthermore, it was found that the upregulation of several Aldo-keto reductases, AKR1C1, AKR1C2, and AKR1C3, protected cells from the ferroptosis persuade by the inhibition of the x_c_^−^ system [35].

The article "Ferroptosis: A Novel Therapeutic Direction of Spinal Cord Injury" was retracted in 2023. Reasons: signs of a paper mill; suspected computer-generated content; unreliable results or conclusions; concerns about the data.

### 3.3. Metabolism of GSH/GPX4 and Regulatory Mechanisms of Ferroptosis

Glutathione peroxidase 4 (GPX4) contributes greatly as an antioxidant in the modulation of ferroptosis. It can reduce complex hydrogen peroxide (e.g., phospholipid hydrogen peroxide and cholesterol hydrogen peroxide) to their respective peroxidation products, thus blocking the chain reaction of lipid peroxidation and consequently inhibiting ferroptosis [36].

The glutamate/cystine antiporter system x_c_^−^ comprises two subunits, namely, SLC3A2 and SLC7A11. Their expression is a potential marker for xCT function and selenoprotein production capacity. They are responsible for the one-on-one transmembrane interchange of cystine out of the cell and intracellular glutamate, and the former is then reduced to cysteine to synthesize glutathione [8, 37]. Glutathione (GSH) is synthesized by three amino acids: cysteine, glycine, and glutamic acid. Glutathione (GSH) is produced by the following amino acids: glycine, cysteine, and glutamic acid. The rate-limiting agent of the GSH reaction is the presence of cysteine. The expression and activity of GPX4 are sustained by GSH due to it being a principal cofactor.

Studies have shown that inhibiting glutathione synthesis to promote its depletion can cause ferroptosis in some cells. For example, in some cellular environments, ferroptosis arises as a result of inhibition of the rate-limiting enzyme, glutamate-cysteine ligase along with buthionine-(S, R)-sulfoximine [38]. In an environment with reduced GSH, GPX4 can convert PLOOH to the corresponding alcohol or free hydrogen peroxide in water, thus breaking the chain reaction of antilipid peroxidation and consequently inhibiting ferroptosis [8, 9]. In addition, GPX4 overexpression can alleviate resibufogenin-induced ferroptosis in colorectal cancer cells [39]. Conversely, in a study, inducible GPx4 inactivation in mice and cells revealed that 12/15-lipoxygenase-derived lipid peroxidation was a specific downstream event that triggered apoptosis-inducing factor- (AIF-) mediated cell death, which could be completely blocked by *α*-tocopherol (a-Toc), 12/15-lipoxygenase inhibitors, or siRNA-mediated AIF silencing [40]; this was confirmed as ferroptosis in follow-up studies.

GPX4 gene-knockout mice display inhibited ferroptosis, which indicates that GPX4 has a vital role in neuroprotection of the cerebellum, hippocampus, and motor neurons [40–43], thus providing a reliable genetic basis for it. In general, when GSH is reduced or depleted or when its synthesis is prevented, the ROS scavenging function of GPX4 is affected. However, the deletion of cysteinyl-tRNA synthetase led to the accumulation of cystathionine, a metabolite of the transsulfuration pathway, and upregulated the genes associated with serine biosynthesis and transsulfuration, which ultimately inhibited cystine deprivation-induced ferroptosis [44]. In the x_c_^−^ system, the expression and activity of SLC7A11 are positively regulated by NFE2L2 [45] and negatively by tumor suppressor genes, such as TP53 [46], BAP1 [47], and BECN1 [48]. This regulatory mechanism affects the synthesis of GSH and the downstream execution of ferroptosis. Type I ferroptosis inducers, such as erastin, sulfasalazine, sorafenib, and glutamate, can reduce cystine intake by inhibiting the x^−^ system, thus resulting in deficiency or depletion of GSH synthesis, which in turn affects the synthesis and activity of GPX4 and promotes ferroptosis [44]. Type II ferroptosis inducers (such as RSL3, ML210, FINO2, RSL3, ML162, and FIN56) can interact with and inactivate GPX4 without depleting glutathione [5, 21].

The article "Ferroptosis: A Novel Therapeutic Direction of Spinal Cord Injury" was retracted in 2023. Reasons: signs of a paper mill; suspected computer-generated content; unreliable results or conclusions; concerns about the data.

A recent study showed that IFN-*γ* released by CD8^+^ T cells downregulated the expression of SLC3A2 and SLC7A11, the two subunits of the glutamate–cysteine antiporter system x^−^, and inhibited cystine uptake, thus inhibiting GPX4 synthesis, promoting lipid peroxidation, and ultimately inducing ferroptosis in tumor cells [49]. This finding suggests that the immune system regulates ferroptosis, thus further complicating the network of regulatory mechanisms of ferroptosis. Furthermore, several non-GPX4 pathways, including AIFM2–CoQ10, GCH1–BH4, and ESCRT-III membrane repair systems, also have a context-dependent role in protection in opposition to oxidative harm during ferroptosis [5].

## 4. Ferroptosis Relation with Other RCDs

### 4.1. Ferroptosis and Apoptosis

To our knowledge, although there is no straight link between ferroptosis and apoptosis, some signs are suggesting that they interact with each other. For example, glutathione deprivation induces not only ferroptosis but also apoptosis and sensitization to apoptosis inducers, such as Smac-mimics [50, 51]. Similarly, GPX4-knockout mice are significantly more delicate than wild-type mice to oxidative stress-induced apoptosis [52]. The depletion of glutathione in the cytoplasm has been suggested to promote ferroptosis, whereas depletion of glutathione in the mitochondria has been suggested to promote apoptosis [53]. If this hypothesis is reasonable, it is worth investigating whether genetic phenotypes altered by GPX4 gene silencing or knockdown induce ferroptosis and apoptosis to the same extent and whether the two cell death pathways are independent.

The article "Ferroptosis: A Novel Therapeutic Direction of Spinal Cord Injury" was retracted in 2023. Reasons: signs of a paper mill; suspected computer-generated content; unreliable results or conclusions; concerns about the data.

In addition, a study on sorafenib with multiple effects found that different cells had different sensitivity to sorafenib. In some cell lines, higher doses of sorafenib could induce apoptosis or other forms of cell death. However, in the same cell line, low-dose sorafenib induced ferroptosis instead of apoptosis [53].

### 4.2. Ferroptosis and Necroptosis

Both ferroptosis and necroptosis have an essential contribution to the disease progression of SCI and other ischemic diseases. Accumulating evidence has suggested that necroptosis and ferroptosis coexist with crosstalk and interaction. Studies imply that both ferroptosis and necroptosis contribute to the advancement of various diseases, including stroke, carcinoma, disorders related to the central nervous system, and chronic obstructive pulmonary disorder [54].

GPX4 is the key protein responsible for the antioxidation of ferroptosis, and we found that GPX4 deficiency not only induced ferroptosis but hematopoietic cells of mice deficient in GPX4 resulted in anaemia owing to the induction of RIP3-dependent necroptosis (but not apoptosis and ferroptosis) [55].

*In vivo*, microscopy imaging showed that ferroptosis simultaneously mediated renal tubular necroptosis and triggered a toxic immune response in the models of ischemia/reperfusion injury and acute renal injury [56]. In another ischemia/reperfusion model, by regulating the ferroptosis-sensitive markers ACSL4 and the necroptosis-sensitive marker mixed lineage kinase domain-like (MLKL), it was found that the ACSL4 deficiency resulted in the increase of MLKL levels and that the loss of MLKL augmented the sensitivity of cells to ferroptosis. This resistance to one RCD pathway causing cell death through another RCD pathway indicates alternate apoptotic modalities are ferroptosis and necroptosis [57].

Neuronal death after hemorrhagic stroke is characterized by both ferroptosis and necroptosis *in vitro* and *in vivo*. The findings revealed increased phosphor-ERK1 (molecular markers of ferroptosis) and mRNA levels of necroptosis markers (RIP1 and RIP3) in hemin-induced cell death. Caspase-dependent apoptosis or autophagy was not identified, and ferroptosis inhibitors (Fer-1, DFO, and Trolox) and necroptosis inhibitors (necrostatin-1) were found to eliminate the lethal toxicity of hemin and haemoglobin [58].

However, the morphological features of hemin-induced ferroptosis were not observed by transmission electron microscopy (TEM), whereas the main features observed were the ultrastructural features of necroptosis, including the disintegration of organelles and the loss of plasma membrane integrity. The exact mechanisms involved are unclear. In organelle microstructures, although the inhibition of mitochondrial complex triggers the increase of mitochondrial autophagy-dependent ROS, thus leading to necroptosis and ferroptosis of melanoma cells [59], the exact mechanism of mitochondrial involvement in ferroptosis remains unclear. 1-Methyl-4-phenylpyridinium (MPP+) can reportedly induce nonapoptotic cell death in the human neuroblastoma cell line SH-SY5Y (a widely used Parkinson's disease model). This mode of cell death is sensitive to both NEC-1 and Fer-1. Interestingly, although MPP+-induced cell death and ferroptosis have some common characteristics and can be inhibited by Fer-1, the mitochondria herein appear swollen rather than shrunk, and shrunk mitochondria are a distinguishing feature of ferroptosis [60]. Recently, a study found that the necroptosis of macrophages induced by *Mycobacterium tuberculosis* infection is associated with the reduced expression of GSH and GPX4 and can be blocked by an iron chelator (PIH) or a lipid peroxidation inhibitor (Fer-1). This result can be extended to an *in vitro* model of necroptosis established by human monocyte-derived macrophages [61].

The article "Ferroptosis: A Novel Therapeutic Direction of Spinal Cord Injury" was retracted in 2023. Reasons: signs of a paper mill; suspected computer-generated content; unreliable results or conclusions; concerns about the data.

### 4.3. Ferroptosis and Autophagy/Ferritinophagy

Several types of selective autophagy have been stated, such as ferritinophagy, clockophagy, lipophagy, mitophagy, and chaperone-mediated autophagy, to contribute to the final execution of ferroptosis by degrading ferroptosis resistance-related proteins or organelles [17]. Ferritinophagy helps initiate ferroptosis by degrading ferritin, which elicits labile iron overload(IO), lipid peroxidation, membrane damage, and the subsequent apoptosis. It is facilitated by a selective cargo receptor, namely, nuclear receptor coactivator 4 (NCOA4), which attaches to ferritin and transfers it to autophagosomes and then to lysosomes to degrade ferritin and release free iron [62, 63]. Its specific inhibitor or inhibition of NCOA4 levels can reduce the sensitivity of different cell lines to ferroptosis [18, 64, 65].

Although there is a biochemical link between NCOA4-mediated ferritinophagy and ferroptosis, current findings have shown a positive correlation among them (i.e., NCOA4- mediated ferritinophagy can induce ferroptosis) [65–67]; therefore, the relationship between remains controversial. For example, NCOA4 levels varied by ferroptosis inducer, with increased expression reported in hepatic stellate cells (HSCs) after sorafenib treatment, no differential expression in pancreatic cancer cells after elastin treatment, and elastin therapy resulted in even lower levels in MEFs or artesunate treatment in HSCs [62]. Unlike in ferroptosis, in rapamycin-induced autophagy, no characteristic morphological features were observed under TEM (e.g., the formation of double-membrane vesicles), and particular inhibitors of autophagy (bafilomycin A1, 3-methyladenine, and chloroquine) did not rescue ferroptosis [6].

The article "Ferroptosis: A Novel Therapeutic Direction of Spinal Cord Injury" was retracted in 2023. Reasons: signs of a paper mill; suspected computer-generated content; unreliable results or conclusions; concerns about the data.

Another recent study showed that NCOA4 deficiency eliminated ferritinophagy, increased ferritin levels, and made cells more durable to elastin but more tactful to RSL3. Further studies revealed that erastin encourages cellular ferritinophagy in an NCOA4-dependent manner, enlarging the intracellular free iron content, lipid peroxidation levels, and sensitivity to ferroptosis. In contrast, RSL3 did not regulate ferritinophagy, while NCOA4 overexpression delayed RSL3-induced cell death indicating that RSL3's mode of action has nothing to do with the ferritin degradation process [64].

The model established with a new ferroptosis inducer Formosan C (FC) also confirmed that ferritinophagy was significantly involved in ferroptosis induced by FC in cells with elevated NCOA4 [68]. Santana-Codina et al. have further elaborated on the mechanisms by which NCOA4 regulates ferroptosis [62]. In addition, the overexpression of ferritin heavy chain 1 (FTH1) can compromise the function of ferritinophagy and downregulate the level of NCOA4, thus inhibiting ferroptosis-induced apoptosis [68, 69]. These findings suggest that the extent of the effect of ferritinophagy on ferroptosis is linked to the specific intra- and extracellular environment and that additional *in vivo* and *in vitro* research may help elucidate the mechanism by which NCOA4 regulates ferroptosis. Furthermore, the data propose that the inhibition of ferroptosis through the regulation of ferritinophagy may herald a probable target for the treatment of some neurological diseases.

## 5. Research Progress of Ferroptosis in SCI

### 5.1. The Current Condition of Spinal Cord Injury Treatment

After spinal cord injury, local tissue destruction is identified by hemorrhage, local IO, demyelination, axonal loss, cell death, immune cell bracing and penetration, and destruction of the blood–spinal cord barrier [78, 79]. These complex pathophysiological changes make it difficult for clinical strategies to precisely regulate the development of cascades. The process of spinal cord injury has been separated into two stages: primary and secondary injuries. The initial stage is the primary injury, which is usually caused by an external mechanical trauma and is often difficult to reverse. In primary injury, injury severity depends primarily on the kinetics and the duration of the compression [78]. With the destruction and disruption of cellular interactions in the spinal cord tissues, including astrocytes, neurons, microglia, and oligodendrocytes, and the onset of biochemical and physiological changes, a series of events culminating in the secondary injury are activated which has been reported to associate with ferroptosis [78, 80].

The article "Ferroptosis: A Novel Therapeutic Direction of Spinal Cord Injury" was retracted in 2023. Reasons: signs of a paper mill; suspected computer-generated content; unreliable results or conclusions; concerns about the data.

Consequently, secondary damage to cells and axons occurs during this period and is exemplified by the production of ROS, ion disorders (including but not limited to Fe^2+^), glutamate-mediated excitotoxicity, and immune-related neurotoxicity [78]. Therefore, it is as important as it is difficult to effectively block and reverse the process of secondary injury.

### 5.2. Potential Drug Targets of Ferroptosis in SCI

As with certain death of cell induced by erasing or RSL3, a series of signature events of ferroptosis occur after spinal cord injury, namely, iron overload, the collection of ROS, and lipid peroxidation at the site of injury; these can be detected by different methods [1, 81]. In the spinal cord, GPX4 is generally considered in the neuronal cytoplasm and the nuclei of oligodendrocyte cells but not in the astrocyte cells [82]. Oligodendrocytes are a type of myelin cells that promote axonal proliferation and myelin sheath formation [83], and astrocytes are a crucial element of the fibrous glial scar that forms around the site of SCI [84].

### 5.3. Valid Models to Evaluate Ferroptosis Treatment in SCI

In the ferroptosis model of oligodendrocytes (OLN-93 cells), which is induced by RSL-3, liproxstatin-1 inhibited the mitochondrial lipid peroxidation, reduced the concentration of ROS and MDA, and restored the expression of GSH, GPX4, and ferroptosis inhibitor protein 1 [71]. Therefore, we speculate that the damage to oligodendrocytes by ferroptosis will exacerbate demyelination after SCI and that liproxstatin-1 will enhance the antioxidant activity of oligodendrocytes and resist ferroptosis by upregulating the level of GPX4 in the nucleus of oligodendrocytes. Thus, it would be interesting to verify the possibility of liproxstatin-1 to restore axonal continuity after SCI by *in vivo* experiments. Similar to this, in a rat model of SCI, mRNA ranks of ferroptosis-related genes, namely, Acyl-CoA synthetase family member 2 (ACSF2) and iron-responsive element-binding protein 2 (IREB2), were significantly upregulated after SCI, and after treatment with DFO, the level of IREB2 and ACSF2 mRNA was dramatically reduced, the survival rate of neurons was improved, the glial proliferation was inhibited, and the expression of GPX4, xCT, and glutathione was significantly increased [22].

The article "Ferroptosis: A Novel Therapeutic Direction of Spinal Cord Injury" was retracted in 2023. Reasons: signs of a paper mill; suspected computer-generated content; unreliable results or conclusions; concerns about the data.

Compared with the first generation ferroptosis inhibitor (Fer-1), intraperitoneal injection of the third-generation ferroptosis inhibitor (SRS16-86) can more stably and effectively upregulate the expression of the anti-ferroptosis factors GPX4, GSH, and xCT and downregulate 4HNE (a marker of lipid peroxidation) by increasing the survival estimate of neurons, reducing the proliferation of astrocytes, and reducing the level of inflammation after SCI to promote functional recovery after SCI [70]. We can interpret from the above data that the rescue effects of GPX4, GSH, and xCT suggest that DFO and SRS16-86 inhibit ferroptosis by increasing the resistance of neurons to toxic lipid oxidation to varying degrees. Glial scars have long been known to constitute a substantial impediment to axonal regeneration. The scars can reportedly promote regeneration as part of the process of endogenous local immune regulation and repair processes [85].

Furthermore, in a mice model of SCI, depriving the scar of astrocyte components has been shown to aggravate the injury and reduce the expression of regenerative components [86]. Therefore, the synthetic inhibition of glial proliferation by DFO and SRS16-86 may involve more complex mechanisms. According to a recent study, the accumulation of iron in the motor cortex increased significantly in a rat model of SCI, thus resulting in the buildup of lipid reactive oxygen species (ROS), which gradually led to ferroptosis of the motor neurons. In addition, activated microglia in the motor cortex secretes rich nitric oxide (NO), which reportedly regulates cellular iron homeostasis-related proteins (IRP1, TfR1, DMT1, and ferritin) and induces IO in motor neurons by changing neuronal iron homeostasis [76].

This suggests that the induction of ferroptosis in the motor cortex may be the reason behind the difficulty in the healing of motor function after SCI. These findings might lead to a novel therapeutic method for SCI. By stimulating the AKT/Nrf2/HO-1 signaling pathway, the anti-inflammatory mediator lipoxin A4 can reduce ferroptosis in spinal cord neurons [77]. Similarly, syringic acid [75], proanthocyanidins [73], and zinc [74] all reversed ferroptosis to varying degrees by activating the Nrf2/HO-1 pathway. It is worth mentioning that Nrf2 is oxidative stress in cells and is regulated by a crucial transcription factor and regulates hundreds of antioxidant genes. So far, Nrf2 controls virtually all of the genetic codes involved in ferroptosis, such as GPX4 and xCT [87]. Further studies of the Nrf2/HO-1 pathway may open new avenues for inhibiting ferroptosis. These data provide a new perspective for us to further understand and regulate ferroptosis in SCI and may give a powerful theoretical basis and therapeutic strategy for the therapy of SCI. Drugs associated with ferroptosis used to treat SCI are shown in Table 1.

The article "Ferroptosis: A Novel Therapeutic Direction of Spinal Cord Injury" was retracted in 2023. Reasons: signs of a paper mill; suspected computer-generated content; unreliable results or conclusions; concerns about the data.

### 5.4. Summary and Outlook

Ferroptosis is a newly discovered mode of RCD and has attracted great interest due to its complexity and heterogeneity. The major focus of this essay is on the key processes of ferroptosis, its role in spinal cord injury, and potential therapeutic possibilities. So far, a lot of progress has been achieved in the field of ferroptosis research. In addition, ferroptosis as an important participant in the spinal cord's secondary phase injury has been confirmed by many reports in the literature. However, the understanding of ferroptosis is still very limited and in the preliminary stage, and many preliminary findings need further verification.

First, the effector molecules of ferroptosis are still unclear. Typical RCDs have their characteristic effector molecules, such as caspases (a marker of apoptosis), MLKL (a marker of necroptosis), LC3-II (a marker of autophagy), and gasdermin D (a marker of pyroptosis) [4, 88]. Although GPX4 is a key antibody to ferroptosis, it not only regulates ferroptosis but also inhibits apoptosis [89] and necroptosis [55], as a response to various tissue damage. Therefore, markers to identify ferroptosis are still lacking.

Secondly, it is still not known how to define the interaction of ferroptosis with other RCDs. In-depth studies on ferroptosis have suggested that ferroptosis shares some of the intermediate signals and molecular regulators with other types of RCDs. For example, lipid peroxidation and regulators of ferroptosis (e.g., SLC7A11) can also regulate other types of RCDs [90, 91]. In addition, the inhibition of ferroptosis may lead to cellular selection to participate in different RCDs' lethal subroutines rather than to avoid cell death; the exact mechanism by which cells are selected and transformed in the lethal program remains unclear.

Finally, the ultimate executor of ferroptosis remains unclear. Although the process of lipid peroxidation and its products promote the cleavage of cell membranes, it may be considered an intermediate event in ferroptosis. The spinal cord comprises different types of cells, and the nervousness of different cell types to ferroptosis after spinal cord injury also needs to be further investigated. Although ferroptosis inhibitors applied to SCI can reduce spinal cord injury to varying degrees and promote recovery of neurological function. These advantages, however, are based mostly on cellular and animal models and have yet to be converted into clinical applications. These questions will inform our next research efforts and lead to a deeper understanding of the potential opportunities of ferroptosis in the treatment of spinal cord injury.

The article "Ferroptosis: A Novel Therapeutic Direction of Spinal Cord Injury" was retracted in 2023. Reasons: signs of a paper mill; suspected computer-generated content; unreliable results or conclusions; concerns about the data.

## Figures and Tables

**Figure 1:** The mechanism of ferroptosis.

**Table 1:** Ferroptosis-associated drugs used to treat SCI. xCT: system x_c_^−^ light chain; GSH: glutathione; GPX4: glutathione peroxidase 4; ACSF2: Acyl-CoA synthetase family member 2; IREB2: iron responsive element-binding protein 2; Nrf2: nuclear factor-erythroid 2-related factor 2; HO-1: heme oxygenase-1; FSP1: ferroptosis inhibitory protein; EGCG, (−)-epigallocatechin-3-gallate; PKD1: protein kinase D1; SOD: superoxide dismutase.

Year	Drugs	Categories	Experimental mode	Potential approach
2019	Deferoxamine [22]	Iron chelator	Rat	Upregulation of xCT, GSH, and GPX4 levels and downregulation of ACSF2 and IREB2 expression
2019	SRS 16-86 [70]	Specific inhibitor	Rat	Upregulation of xCT, GSH, and GPX4 levels
2020	Liproxstatin-1[71]	Lipid peroxidation inhibitor	Cell	Upregulation of GSH, GPX4, and FSP1 levels
2020	EGCG [72]	Lipid peroxidation inhibitor	Cell +rat	Upregulation of PKD1Phosphorylation levels
2020	Proanthocyanidin [73]	Lipid peroxidation inhibitor	Mice	Upregulation of GSH, GPX4, Nrf2, and HO-1 levels, chelated iron
2021	Zinc [74]	Lipid peroxidation inhibitor	Mice	Upregulate the expression of NRF/HO-1, increase the levels of GSH, GPX4, and SOD, and downregulate the level of lipid iron
2021	Carnosic acid [75]	Lipid peroxidation inhibitor	Cell	Upregulation of Nrf2, GSH, and GPX4 levels
2021	Ferrostatn-1 [76, 77]	Lipid peroxidation inhibitor	Cell	Upregulation of GSH and GPX4 levels and downregulation of lipid peroxidation
2021	Lipoxin A4 [77]	Specific inhibitor	Cell	Activation of Akt/Nrf2/HO-1 pathway

## Data Availability

The data used to support this study is available from the corresponding author upon request.
